# Intra-Articular Injection of PRP in the Treatment of Knee Osteoarthritis Using Big Data

This article has been retracted.

**DOI:** 10.1155/2021/4504155

**Published:** 2021-10-26

**Authors:** Zhijin Lin, Ling He

**Affiliations:** ^1^Xingtai People's Hospital, Doctor–Patient Communication Office, Xingtai 054001, China; ^2^Hebei Eye Hospital, Otolaryngology Head and Neck Surgery, Xingtai 054001, China

## Abstract

Observing data on the characteristics of intra-articular injection of sodium citrate for knee osteoarthritis is an important reference value for human safety and evacuation design. To address the problems of slow data collection and poor accuracy of results of knee osteoarthritis behavior, under intensive conditions of intra-articular injection for knee osteoarthritis, this paper designs a data mining-based feature extraction system for intra-articular injection of sodium citrate for knee osteoarthritis. Using the Hadoop architecture, we extract the basic data of human behavior in the two-dimensional plane by storing and stitching the collected continuous data and discriminate the behavioral categories of knee osteoarthritis. We collected a real dataset from 84 patients with knee osteoarthritis treated in our hospital from October 2019 to October 2020. The dataset was divided into 42 patients in the tretinoin group and 42 patients in the sodium glutamate group according to the randomized number table method. The trimethoprim group was treated with intra-articular injection of trimethoprim, and the sodium citrate group was treated with intra-articular injection of sodium citrate. The clinical efficacy, joint mobility, intra-articular fluid volume, Lysholm score of knee joint, numerical pain intensity scale (NRS) score, and adverse effects of the two groups were compared before and after treatment. In our experiments, we observed that, compared with triamcinolone acetonide intra-articular injection, sodium hyaluronate intra-articular injection is more effective in the treatment of knee osteoarthritis. It can effectively improve knee function and reduce pain and adverse reactions.

## 1. Introduction

Knee osteoarthritis is a disease based on degenerative pathological changes [1, 2]. Intra-articular injection of tretinoin is often used clinically for the treatment of knee osteoarthritis, but the incidence of adverse effects is high, the efficacy of the drug is insufficient to control disease progression [3], and the overall efficacy is poor. The study studied the intra-articular injection of sodium glutamate for the treatment of knee osteoarthritis. Artificial intelligence (AI) is a concept of using computers to construct complex machines with the same essential characteristics as human intelligence. Machine learning refers to the use of algorithms to help make decisions to complete intelligent tasks and is a method to achieve artificial intelligence, while deep learning is developed in recent years thanks to the accumulation of big data, relying on neural network models, a technology to achieve machine learning [3, 4].

In fact, the theory of AI has been proposed for half century, and the idea of machine learning can be traced back to the 1980s, while the real rapid development of deep learning has started from the establishment of various open-source labeled image data materials since 2010. Currently, deep learning mainly consists of computer vision and natural language processing. The purpose of this paper is to introduce AI in orthopedic applications, and to some extent, the prospect of computer vision and medical imaging technologies and artificial neural networks in orthopedic applications [5]. In orthopedic imaging data, we mainly target problems including fracture, spinal degeneration and deformity, and joint disorders. And most of these problems have distinct features that are well suited for the application of AI. For example, for the judgment of fracture, normal skeletal bone is continuous, and the learning of skeletal image signals in massive images can empower the model to quickly detect fractures, and even for tiny fracture signs that are easily missed, the model can screen them out in seconds. In 2018 model development experiments that pooled 130,000 flat skeletal films of the limbs, the sensitivity of fracture diagnosis reached 80.8% in the diagnostic manual pure group and the intelligent assisted group, respectively [6].

The PRP injection therapy has many advantages: first, PRP is autogenous, without the risk of disease transmission and immune rejection, which is safe and effective. PRP has been used in many countries and is widely used in many disciplines. In Europe and the United States, especially, many famous athletes such as golf star Tiger Woods, tennis star Rafael Nadal, and basketball star Kobe Bryant, have received PRP treatment several times for knee sprains and chronic tendon injuries [7, 8]. PRP has been widely used in the field of bone and joint diseases and soft tissue injuries, including degenerative osteoarthritis (knee, ankle, hip, etc.), articular cartilage injuries, tendon, and ligament injuries (rotator cuff injury, Achilles' tendon injury, patellar tendon injury, tennis elbow, golf elbow), and muscle injuries. A schematic diagram of human joints is shown in Figure 1.

Although hypertonic acid can improve cartilage lubrication and relieve pain, this therapy cannot fundamentally restore the function of knee cartilage. In contrast to traditional treatments such as hypertonic acid injections, the platelets and various growth factors in PRP accelerate the process of tissue recovery, reduce pain and control inflammation through self-regulation and repair, and can achieve the function of repairing damaged tissues [9, 10]. PRP has been gradually carried out in orthopedics, rehabilitation, and burns departments in many hospitals in China, with efficacy in the fields of bone disease, trauma, and sports injuries.

Observation of data on the characteristics of intra-articular injection of sodium nitrate for knee osteoarthritis is an important reference value for human safety and spring design. To address the problems of slow data collection and poor accuracy of results of knee osteoarthritis behavior under intensive conditions of intra-articular injection for knee osteoarthritis, this paper designs a data mining-based feature extraction system for intra-articular injection of sodium nitrate for knee osteoarthritis. Using the Hadoop architecture, we extract the basic data of human behavior in the two-dimensional plane by storing and stitching the collected continuous data and discriminate the behavioral categories of knee osteoarthritis. Eighty-four patients with knee osteoarthritis treated in our hospital from October 2019 to October 2020 were divided into 42 patients in the tretinoin group and 42 patients in the sodium glutamate group according to the randomized number table method. The trimethoprim group was treated with intra-articular injection of trimethoprim, and the sodium nitrate group was treated with intra-articular injection of sodium nitrate. The clinical efficacy, joint mobility, intra-articular fluid volume, Lysholm score of knee joint, numerical pain intensity scale (NRS) score, and adverse effects of the two groups were compared before and after treatment. The major contributions of our paper are highlighted as follows:

1. This paper designs a data mining-based feature extraction system for intra-articular injection of sodium citrate for knee osteoarthritis
2. Using the Hadoop architecture, we extract the basic data of human behavior in the two-dimensional plane by storing and stitching the collected continuous data
3. discriminate the behavioral categories of knee osteoarthritis

The reminder of this paper is organized as follows. In Section 2, we introduce the core technology of the feature extraction system. In Section 3, we present the system validation. In Section 4, we describe the PRP case sharing. In Section 5, we discuss materials and method. In Section 6, we explain our findings. Finally, we conclude the paper in Section 7.

## 2. The Core Technology of the Feature Extraction System

The data extraction of vitreous acid sodium intra-articular injection for knee osteoarthritis, which contains the extraction of basic data of osteoarthritis of the spliced knee, the discrimination of the type of knee osteoarthritis, and the extraction of characteristic parameters of traffic behavior, is the core part of the knee osteoarthritis feature extraction system, which transforms a large amount of video data into the form of resultant data records.

### 2.1. Multicamera Video Stitching

Video switching is essentially the stitching of video frame images using image stitching algorithms to process video sequences. Video image stitching mainly includes image alignment (feature point extraction and feature matching) and image fusion 2 steps. The video stitching process is shown in Figure 2.

#### 2.1.1. SIFT Feature Point Extraction

The feature points of the sample knee osteoarthritis image and the target knee osteoarthritis image are extracted in the following steps. Extract the polar points in the Gaussian differential scale space of the knee osteoarthritis image to obtain scale invariance; determine the feature points by fitting function and remove the unstable polar points; then, within the neighborhood window centered on the feature points, use the gradient direction histogram to count the gradient direction of pixels in the neighborhood and divide the 360° circle into 36 columns by 10°; the length of the columns represents the magnitude of the gradient, and the histogram. The direction of the peak column is the main direction of the gradient in the neighborhood of the feature point, and the gradient direction larger than 80% of the peak of the main direction can be used as an auxiliary direction to increase the robustness of the detection point; finally, a 128-dimensional feature descriptor is generated according to the change of the points around the feature point [8].

#### 2.1.2. Feature Matching

After obtaining the feature points of the two knee osteoarthritis images, the Euclidean distance was used as a metric to match the feature points of the two images. The closest and second closest feature points of the sample image were found out, and the ratio of the closest and second closest distance was found out, and the pair of feature points was formed when it was less than a certain threshold. The random sample consensus (RANSAC) algorithm is used to remove the wrong matching pairs and improve the accuracy [11].

#### 2.1.3. Image Fusion

To make the transition of overlapping regions more perfect, a nonlinear weighted fusion method is used to fuse the knee osteoarthritis images. The key frames of the knee osteoarthritis video were extracted, and multiple key frames were repeated to complete the video switching.

### 2.2. Basic Data Extractions for Knee Osteoarthritis

To extract the basic knee osteoarthritis data, the target knee osteoarthritis is first detected from the stitched top video, then the knee osteoarthritis motion trajectory is extracted based on the motion of the target knee osteoarthritis center of mass, and finally the knee osteoarthritis time and position coordinates are extracted based on the knee osteoarthritis motion trajectory and the basic knee osteoarthritis dataset is generated [12, 13].

#### 2.2.1. Knee Osteoarthritis Detection

The osteoarthritis detection of knee joint is achieved by interframe differential method for the captured knee osteoarthritis video. The default 1 s is 24 frames, and the frames are selected at 1 s interval, so the nth frame and the *n*th + 24 the frame of the knee osteoarthritis video sequence are *f*_*n*_ and *f*_*n*+24_, and the gray scale values of the corresponding pixel points of the two frames are subtracted and their absolute values are taken to obtain the difference image *D*_*n*_. The threshold *T* is set to minimize each pixel point in *D*_*n*_ (when the pixel point in 55 is greater than or equal to *T*, the pixel value of that point is 255, which is the motion target point). When the pixel point in *D*_*n*_ is greater than or equal to *T*, the pixel value of this point is 255, which is the motion target point; when the pixel point in 55 is less than *T*, the pixel value of this point is 0, which is the background point). Finally, we obtain the finalized image *R*_*n*_.

#### 2.2.2. Knee Osteoarthritis Trajectory Extraction

The center of mass of the knee osteoarthritis target in the minimized image containing the knee osteoarthritis target is used as the reference point of the motion trajectory, and after calculating the center of mass of the knee osteoarthritis target, the video is superimposed on multiple frames, and the motion trajectory of the knee osteoarthritis can be obtained by connecting the calculated center of mass of the knee osteoarthritis target in turn.

#### 2.2.3. Data Extraction Based on Knee Osteoarthritis

A plane right-angle coordinate system is established at each node facility of the station with the main flow direction of knee osteoarthritis as the *y*-axis, and the position coordinates (*x*, *y*) dataset corresponding to the moment of knee osteoarthritis movement *t* is obtained after coordinating the position of knee osteoarthritis.

### 2.3. Determination of Knee Osteoarthritis Category and Extraction of Characteristic Parameters

Before extracting the characteristic parameters of knee osteoarthritis, it is necessary to judge the traffic behavior category according to the indicators of knee osteoarthritis: passage space, speed, displacement, and distance. Therefore, on the basis of extracting time and location data, the behavior judgment indicators are calculated first to form a behavior judgment dataset, and the characteristic parameters are calculated after subsequent calls to this dataset for behavior category judgment.

#### 2.3.1. Category Judgment

Based on the kinetic theory of knee osteoarthritis, intra-articular injection of sodium nitrate for the treatment of knee osteoarthritis was classified into three categories of single-unit behavior, interaction behavior, and obstacle avoidance behavior according to the individual's individual action, coupling action between individual and individual, and coupling action between individual and obstacle [14]. The three types of behaviors were subdivided into walking behavior, wandering behavior, and staying behavior; interaction behavior was divided into following behavior, overtaking behavior, avoidance behavior, and insertion behavior; and obstacle avoidance behavior was divided into changing path behavior and backward behavior. To extract the characteristic parameters of knee osteoarthritis more efficiently, the knee osteoarthritis behavior category can be judged in advance. In addition, since single-unit behavior or interaction behavior will exist at the same time of obstacle avoidance behavior, the obstacle avoidance behavior discrimination is carried out simultaneously with single-unit behavior and interaction behavior discrimination. The process of single-unit behavior and interaction behavior discrimination for knee osteoarthritis is shown in Figure 3. The process of obstacle avoidance in knee osteoarthritis is shown in Figure 4.

#### 2.3.2. Feature Parameter Extraction

After judging the knee osteoarthritis category, the behavioral feature parameters are extracted according to the basic dataset and the feature parameter calculation formula. For example, the dwell behavior feature parameters include knee osteoarthritis speed, dwell range and dwell time; the following behavior feature parameters include following speed difference, lateral spacing, following distance and speed direction angle; the lane-changing behavior feature parameters include the amount of change of knee osteoarthritis travel direction, the longitudinal distance between the starting point of knee osteoarthritis lane-changing behavior and the center of the obstacle and knee osteoarthritis cumulative lateral shift distance [15, 16].

## 3. System Validation

### 3.1. Following Behavior Features Parameter Extraction

The video of knee osteoarthritis in our hospital was collected, and the feature extraction system based on video data mining of sodium glacial intra-articular injection for knee osteoarthritis was compared with the feature parameters of osteoarthritis following behavior of the knee joint obtained by manual calculation to verify the validity of the data. A two-dimensional right-angle coordinate system was established at the gate, and the trajectory of knee osteoarthritis following behavior is shown in Figure 5. The video is playing at 4 frames/s.

(3) $$\begin{array}{c} d_{ij}=\sqrt{{\left(x_{jm}-x_{im}\right)}^{2}+{\left(y_{jm}-y_{im}\right)}^{2}}, \end{array}$$

Following behavior refers to the behavior of following the knee osteoarthritis in front of the knee osteoarthritis by changing the walking path and walking speed during the walking process under the influence of other knee osteoarthritis or obstacles within the field of view in a certain density knee osteoarthritis environment. The characteristic parameters of the following behavior are calculated as follows:

(1) $$\begin{array}{c} \Delta V=\left\|{\overset{⟶}{V}}_{i}|-|{\overset{⟶}{V}}_{j}\right\|, \end{array}$$

where Δ*V* is the difference of following velocity, m/s; *V*_*i*_ and *V*_*j*_ are the velocities of follower *i* and follower *j* at the same moment, m/s, respectively.

(2) $$\begin{array}{c} D_{H}=\left|x_{im}-x_{jm}\right|, \end{array}$$

where *D*_*H*_ is the lateral spacing, *m*; *x*_*im*_ and *x*_*jm*_ are the horizontal coordinates of knee osteoarthritis *i* and knee osteoarthritis *j* at time *m*, respectively.where *x*_*jm*_ and *x*_*im*_ are the vertical coordinates of knee osteoarthritis *i* and knee osteoarthritis *j* at time *m*.

(4) $$\begin{array}{c} \theta_{ij}=\arccos\left(\frac{{\overset{⟶}{V}}_{i}\cdot {\overset{⟶}{V}}_{j}}{\left|{\overset{⟶}{V}}_{i}\right|-\left|{\overset{⟶}{V}}_{j}\right|}\right), \end{array}$$

where *v*__*i*__ and *v*_*j*_ are the velocity vectors of knee osteoarthritis *i* and knee osteoarthritis *j* at the same moment, m/s, respectively.

### 3.2. Validation of the Follow-Behavior Feature Parameters

Comparing the system extraction results of knee osteoarthritis following behavior feature parameters with the manual calculation results in Xujing East Station of Shanghai Railway Line 2, the validity of knee osteoarthritis following behavior feature parameters extraction results are verified as shown in Figure 5. Since the system tracks the knee osteoarthritis trajectory with the top of the knee osteoarthritis head as the tracking object, a slight movement of the knee osteoarthritis head will be recognized as a knee osteoarthritis movement, but the knee osteoarthritis is standing still, so there is a slight fluctuation of the system extracted result curve in Figure 6.

As can be seen in Figure 6(a), the lateral distance *D*_*H*_ between the knee osteoarthritis decreases gradually to 0 and the knee osteoarthritis *j* follows the knee osteoarthritis *i* in a forward direction. The difference in following speed Δ*V* and following distance *d*_*ij*_ between the two persons in Figures 6(b) and 6(c) first increases and then decreases because when the followed knee osteoarthritis decelerates and walks to the gate to stop and swipe the card. The following knee osteoarthritis stays in place and then walks toward the followed knee osteoarthritis at a certain speed. As the distance between the two persons decreases, the following knee osteoarthritis gradually decelerates until the two persons maintain normal knee osteoarthritis. Arthritis static spatial requirements of the distance are shown in Figure 6(d). The angle between the following knee osteoarthritis and the followed knee osteoarthritis travel speed *θ*_*ij*_ gradually decreases to 0, and the following knee osteoarthritis changes its travel direction gradually in the same direction as the followed knee osteoarthritis. *t* = 2 s; the abrupt inflection point of the system extraction results is caused by the slight backward movement of the following knee osteoarthritis head as the knee osteoarthritis movement when the knee osteoarthritis is tracked. This is largely caused by the movement of the osteoarthritis in the knee.

Through the previously mentioned validation results, as shown in Figures 6(e) and 6(f), the system extraction results have some errors compared with the manual calculation results but in general meet the actual work requirements and can further optimize the system data mining method to reduce the errors by cleaning the invalid data such as the abrupt inflection point serval data like the angle between the following knee osteoarthritis and the followed knee osteoarthritis walking speed.

## 4. The PRP Case Sharing

Ms. He, aged 45, was admitted to the hospital at 10:43 a.m. on December 29, 2020, with “*pain in both knees for three years*, *aggravated for one month*.” The patient complained of pain in both knees with no obvious cause three years ago, with intermittent attacks. The right knee MRI showed the following: (i) osteophytes in the right knee, (ii) small amount of fluid in the right knee joint cavity and suprapatellar bursa, (iii) bone marrow edema in the right upper tibia, (iv) degeneration of the posterior horn of the medial meniscus and the anterior horn of the lateral meniscus in the right knee, (v) edema of the soft tissue around the right knee, and (vi) degeneration of the anterior cruciate ligament of the right knee (the patient was given trimethoprim injection). After a detailed examination, Dr. Huang Li Eyi, the chief physician of our department, considered the patient's knee injury and suggested the patient have PRP injection treatment, as shown in Figure 7.

## 5. Materials and Methods

### 5.1. General Information

Eighty-four patients with knee osteoarthritis treated at the First People's Hospital of Guangshui City, Hubei Province, from October 2017 to October 2018, were selected and divided into 42 cases in the tretinoin group and the sodium glacial group according to the random number table method. There were 20 cases in the tretinoin group and 22 cases in the female group: ages 37–68 (49.09 ± 9.33) years; duration of disease 4–9 (6.16 ± 2.83) years. The difference between the two groups in terms of gender, age, and disease duration was not statistically significant (as illustrated by the *P* value that is >0.05) and was comparable. The study was supported and approved by the hospital ethics committee, and the patients and their families gave informed consent and signed the informed consent form.

### 5.2. Selection Criteria

Inclusion criteria are as follows: (1) diagnosed knee osteoarthritis [4]; (2) symptoms such as swelling and pain in the knee joint, pain in going up and down stairs, swelling, popping, and fluid accumulation; (3) physical examination and x-ray examination; (4) patients with good self-awareness and mental status; (5) no allergy to tretinoin and sodium nitrate. Exclusion criteria are as follows: (1) patients with malignant tumors or immune system diseases; (2) patients who cannot physically tolerate tretinoin or sodium nitrate treatment; (3) patients with psychiatric diseases.

### 5.3. Treatment Method

The trimethoprim group was treated with trimethoprim acetate injection (Shanghai General Pharmaceutical Co., Ltd., GMP H31021291) 40 mg using intra-articular injection once a week. The vitreous acid sodium group was treated with vitreous acid sodium injection (Shanghai Jingfeng Pharmaceutical Co., Ltd., State Drug Administration H20000643) 25 mg using intra-articular injection once a week. Both groups were treated continuously for five weeks.

### 5.4. Observation Indexes and Methods

We compared the two groups in terms of (1) the clinical efficacy, (2) the joint mobility and the amount of intracellular fluid, and (3) the Lysholm scale score of the knee joint. The Lysholm scale of knee joint [5] included eight evaluation items: pain (25 points), instability (25 points), atresia (15 points), swelling (10 points), limp (5 points), stair climbing (10 points), squatting (5 points), and use of support (5 points), and the total score was 100 points. (4) NRS score of the two groups was compared, and the NRS score ranged from 0 to 10. The NRS score ranges from 0 to 10.0: no pain; 1 to 3: mild pain and tolerable; 4 to 6: severe pain and tolerable; 7 to 10: severe pain and unbearable [6]. The higher the score, the more intense the pain. (5) We compared the adverse effects of the two groups, including gastrointestinal irritation, psychiatric symptoms, and joint edema.

### 5.5. Efficacy Evaluation Criteria

*Significantly Effective.* Symptoms such as knee swelling and pain, walking up and down stairs, swelling, popping and fluid accumulation improved significantly, and the related indexes of clinical x-ray examination improved by more than 80%. *Effective.* Symptoms such as knee swelling and pain, walking up and down stairs, swelling, popping, and fluid accumulation improved, and the related indexes of clinical x-ray examination improved by 30% to 79%. *Ineffective.* Symptoms such as knee swelling and pain, walking up and down stairs, swelling, popping, and fluid accumulation improved by less than 30%. *No Effect.* No improvement or worsening of symptoms such as knee pain, walking up and down stairs, swelling, popping, and fluid accumulation and less than 30% improvement in clinical x-ray indexes. Total effective rate = (effective + effect)/total number of cases × 100%.

### 5.6. Statistical Methods

SPSS 17.0 was used for data analysis. The datum was analyzed by SPSS 17.0.

### 5.7. Results and Discussion

The total effective rate in the sodium nitrate group was 95.24%, which was higher than the 73.81% in the trimethoprim group (*χ*2 = 7.372, *P*=0.007). See Table 1.

### 5.8. Comparison of Joint Mobility and Intracellular Fluid Volume before and after Treatment

Before treatment, there was no statistically significant difference between the two groups in terms of joint mobility and intracellular fluid volume (*P* > 0.05). After treatment, joint mobility and intracellular fluid volume were better in both groups than before treatment, and the sodium nitrate group was better than the tretinoin group (*P* < 0.01). See Table 2.

### 5.9. Comparison of Knee Lysholm Scale Scores before and after Treatment

Before treatment, there was no statistically significant difference between the Lysholm scale scores of knee joints of the two groups (*P* > 0.05). After treatment, the Lysholm scale scores of knee joints of the two groups were significantly higher, and the vertex group was higher than the tretinoin group (*P* < 0.01). See Table 3.

Before treatment, the difference between the NRS score of the two groups was not statistically significant (*P* > 0.05). After treatment, NRS score of the two groups was significantly lower, and the vertex group was lower than the tretinoin group (*P* < 0.05). See Table 4.

The overall incidence of adverse reactions was 7.14% in the sodium nitrate group, which was lower than that of 23.81% in the tretinoin group (*x*^2^ = 4.459, *P*=0.035). See Table 5.

## 6. Discussion

In recent years, the incidence of knee osteoarthritis has been rapidly increasing, which has attracted increasing clinical attention [7]. Patients with knee osteoarthritis are often associated with knee swelling, pain, popping, fluid accumulation, etc. [8]. If left untreated, as the disease progresses, complications such as knee deformity and muscle atrophy will be induced [9], resulting in restricted joint movement and seriously affecting the quality of life. Trimethoprim is an adrenocorticotropic hormone [10], which has strong anti-inflammatory effect but no antibacterial effect [11], can reduce the body's ability to resist infection, and make the body resist disease. Its long-term use is likely to lead to disorders of water, salt, sugar, protein, and fat metabolism, increasing the incidence of adverse reactions and leading to a decrease in drug efficacy. In recent years, intra-articular injection of sodium nitrate has been effective in the treatment of knee osteoarthritis. The intra-articular injection of high molecular weight, concentration, and viscoelasticity of sodium nitrate can significantly improve the inflammatory reaction of synovial fluid. It can increase the content of sodium nitrate in synovial fluid, which can enhance the viscosity and lubricating function of synovial fluid. As a result, it protects articular cartilage, promotes the healing and regeneration of articular cartilage, and slows down the progression of osteoarthritis. The osteoarthritis plays an important role in the progression of many diseases [12].

The results and findings obtained from this study showed that the overall efficiency of the sodium nitrate group was higher than that of the tretinoin group. After treatment, the joint mobility and the amount of intracellular fluid were better in both groups than before treatment, and the sodium nitrate group was better than the tretinoin group. The overall incidence of adverse reactions was lower in the vitreous acid group than in the tretinoin group. The clinical effect of intra-articular injection of sodium nitrate in the treatment of knee osteoarthritis was proved to be good, which can effectively improve the function of the knee joint and reduce the pain of the patients with few adverse effects and can be promoted.

## 7. Conclusions and Future Work

Observation of data on the characteristics of intra-articular injection of sodium nitrate for knee osteoarthritis is an important reference value for human safety and spring design. To address the problems of slow data collection and poor accuracy of results of knee osteoarthritis behavior under intensive conditions of intra-articular injection for knee osteoarthritis, this paper designs a data mining-based feature extraction system for intra-articular injection of sodium nitrate for knee osteoarthritis. By using Hadoop architecture, we store and stitch the collected continuous data, extract the basic data of human behavior in two-dimensional plane, and discriminate the behavior category of knee osteoarthritis. Ultrasound-guided PRP injection therapy yields more intuitive results because platelet plasma is injected directly into the lesion area under ultrasound guidance. Compared with conventional palpation-guided or radiation-guided treatment, ultrasound-guided treatment has the advantages of being real-time, convenient, precise, minimally invasive, economical, and radiation-free. Because of its real-time dynamic observation, ultrasound-guided treatment can help clinicians avoid damage to peripheral nerves, control drug dosage, reduce vascular complications, improve pain, and increase postoperative patient satisfaction.

Using real data collected from 84 patients with knee osteoarthritis treated in our hospital from October 2019 to October 2020, we observed that, compared with triamcinolone acetonide intra-articular injection, sodium hyaluronate intra-articular injection is more effective in the treatment of knee osteoarthritis. It can effectively improve the knee function, reduce pain, and reduce adverse reactions. In the future, where many healthcare costs are borne by the patient, PRP (due to its endogenous production) may aid in lowering the total cost of therapy. It may also accomplish this by reducing the need for painkillers, hospital visits, and surgical intervention. In future, we will more deeply study the impact of our outcomes using huge data from different patients with various parameters and characteristics.

## Figures and Tables

**Figure 1:** Schematic diagram of human joints.

**Figure 2:** Video splicing process.

**Figure 3:** Flow of discrimination between single and interactive behaviors in osteoarthritis of the knee joint.

**Figure 4:** Flow of discriminating behavior of knee osteoarthritis avoidance.

**Figure 5:** Trajectory of knee osteoarthritis following behavior.

**Figure 6:** Validation of the results of extracting the parameters of the knee joint osteoarthritis following behavior features. (a) Lateral distance, (b) transverse spacing, (c) transverse spacing, (d) following speed difference, (e) following distance, and (f) included angle in speed direction.

**Figure 7:** The human joint detection.

**Table 1:** Comparison of the clinical efficacy of the two groups cases (%).

Group	Number of cases	Remarkable effect	Effective	Invalid	Total effective rate (%)
Triamcinolone acetonide formation	42	20 (47.62)	11 (26.19)	11 (26.19)	73.81
Sodium hyaluronate group	42	27 (64.29)	13 (30.95)	2 (4.76)	95.24

Compared with the total effective rate in the tretinoin group, *a*_*p*_ < 0.01.

**Table 2:** Comparison of joint mobility and intracellular fluid volume before and after treatment in the two groups ($\bar{x}\pm s$).

Group	Time	Joint mobility (°)	Intraluminal effusion (°)
Triamcinolone acetonide formation (*n* = 42)	Before treatment	57.28 ± 12.34	6.24 ± 1.09
	After treatment	72.11 ± 13.09	5.22 ± 1.13
Sodium hyaluronate group (*n* = 42)	Before treatment	56.33 ± 12.26	6.19 ± 1.11
	After treatment	85.26 ± 14.14	3.01 ± 1.14
*T*/*P* triamcinolone acetonide group (before and after treatment)		5.343/0.001	4.210/0.001
*T*/*P* sodium hyaluronate group (before and after treatment)		10.018/0.001	12.953/0.001
*T*/*P* value between groups (after treatment)		4.423/0.001	8.923/0.001

**Table 3:** Comparison of Lysholm scale score of knee joint before and after treatment in the two groups ($\bar{x}\pm s$, score).

Group	Number of cases	Before treatment	After treatment	*T* value	*P* value
Triamcinolone acetonide formation	42	49.37 ± 8.03	71.11 ± 10.09	10.926	0.001
Sodium hyaluronate group	42	48.46 ± 8.11	85.27 ± 11.34	17.111	0.001
*T* value		0.517	6.046		
*P* value		0.607	0.001		

**Table 4:** Comparison of NRS scores before and after treatment between the two groups ($\bar{x}\pm s$, score).

Group	Number of cases	Before treatment	After treatment	*T* value	*P* value
Triamcinolone acetonide formation	42	8.37 ± 1.84	5.78 ± 1.67	7.317	0.001
Sodium hyaluronate group	42	8.41 ± 1.76	3.05 ± 1.13	16.608	0.001
*T* value		0.102	8.774		
*P* value		0.919	0.001		

**Table 5:** Comparison of the occurrence of adverse reactions in the two groups (cases (%)).

Group	Number of cases	Gastrointestinal irritation	Mental symptoms	Joint edema	Total incidence (%)
Triamcinolone acetonide formation	42	2 (4.76)	4 (9.52)	4 (9.52)	23.81
Sodium hyaluronate group	42	1(2.38)	1 (2.38)	1 (2.38)	7.14

Comparison with the total incidence in the tretinoin group, *a*_*p*_ ＜ 0.05.

## Data Availability

The datasets used and analyzed during the current study are available from the corresponding author upon reasonable request.
